# Wasp venom peptide improves the proapoptotic activity of alendronate sodium in A549 lung cancer cells

**DOI:** 10.1371/journal.pone.0264093

**Published:** 2022-02-24

**Authors:** Nabil A. Alhakamy, Solomon Z. Okbazghi, Mohamed A. Alfaleh, Wesam H. Abdulaal, Rana B. Bakhaidar, Mohammed O. Alselami, Majed AL Zahrani, Hani M. Alqarni, Adel F. Alghaith, Sultan Alshehri, Shaimaa M. Badr-Eldin, Hibah M. Aldawsari, Omar D. Al-hejaili, Bander M. Aldhabi, Wael A. Mahdi

**Affiliations:** 1 Department of Pharmaceutics, Faculty of Pharmacy, King Abdulaziz University, Jeddah, Saudi Arabia; 2 Advanced Drug Delivery Research Group, Faculty of Pharmacy, King Abdulaziz University, Jeddah, Saudi Arabia; 3 Center of Excellence for Drug Research and Pharmaceutical Industries, King Abdulaziz University, Jeddah, Saudi Arabia; 4 Mohamed Saeed Tamer Chair for Pharmaceutical Industries, King Abdulaziz University, Jeddah, Saudi Arabia; 5 Global Analytical and Pharmaceutical Development, Alexion Pharmaceuticals, New Haven, Connecticut, United States of America; 6 Vaccines and Immunotherapy Unit, King Fahd Medical Research Center, King Abdulaziz University, Jeddah, Saudi Arabia; 7 Department of Biochemistry, Faculty of Science, Cancer and Mutagenesis Unit, King Fahd Medical Research Center, King Abdulaziz University, Jeddah, Saudi Arabia; 8 Centre for Artificial Intelligence in Precision Medicines, King Abdulaziz University, Jeddah, Saudi Arabia; 9 Department of Pharmaceutics, College of Pharmacy, King Saud University, Riyadh, Saudi Arabia; 10 Department of Pharmaceutical Sciences, College of Pharmacy, Almaarefa University, Ad Diriyah, Saudi Arabia; 11 Department of Pharmaceutics and Industrial Pharmacy, Faculty of Pharmacy, Cairo University, Cairo, Egypt; Laurentian University, CANADA

## Abstract

**Background:**

Lung cancer in men and women is considered the leading cause for cancer-related mortality worldwide. Anti-cancer peptides represent a potential untapped reservoir of effective cancer therapy.

**Methodology:**

Box-Behnken response surface design was applied for formulating Alendronate sodium (ALS)-mastoparan peptide (MP) nanoconjugates using Design-Expert software. The optimization process aimed at minimizing the size of the prepared ALS-MP nanoconjugates. ALS-MP nanoconjugates’ particle size, encapsulation efficiency and the release profile were determined. Cytotoxicity, cell cycle, annexin V staining and caspase 3 analyses on A549 cells were carried out for the optimized formula.

**Results:**

The results revealed that the optimized formula was of 134.91±5.1 nm particle size. The novel ALS-MP demonstrated the lowest IC50 (1.3 ± 0.34 μM) in comparison to ALS-Raw (37.6 ± 1.79 μM). Thus, the results indicated that when optimized ALS-MP nanoconjugate was used, the IC50 of ALS was also reduced by half. Cell cycle analysis demonstrated a significantly higher percentage of cells in the G2-M phase following the treatment with optimized ALS-MP nanoconjugates.

**Conclusion:**

The optimized ALS-MP formula had significantly improved the parameters related to the cytotoxic activity towards A549 cells, compared to control, MP and ALS-Raw.

## Introduction

Cancer refers to a group of diseases in which cells proliferate abnormally and spread to surrounding cells and tissues [1, 2]. Its development is associated with numerous risk factors as family history, race, abnormalities in genetics, sex, obesity, bad nutrition, exposure to radiation and stress [3, 4]. Cancer has emerged lately as the world’s second leading cause of death following cardiovascular-related diseases [5]. Importantly, its incidence rate has risen over the last few decades [6, 7]. As a result, innovations and advances in cancer screening, diagnosis, and treatment are fundamentally required. In particular, lung cancer is the leading cause for cancer-related deaths in the world [8, 9]. Over the last century, lung cancer has become an epidemic due to the consistent and dramatical increase in its incidence and death rates, both in men and women [9]. Despite the fact that the ideal chemotherapeutic agent requires direct and continuous administration to the target tumor tissue to maximize the cytotoxic effect to overcome low drug bioavailability occurs at tumor tissue after systemic administration [10–12].

Complementary and alternative medicine refers to medical systems and therapies which are based on skill, knowledge, and practices, theories, philosophies, and the experiences used for maintaining and improving health and for prevention, diagnosis, or treatment of various physical and mental disorder [13]. In this respect, anti-cancer peptides are regarded potential untapped reservoir of effective cancer therapy [14]. They are small polypeptides consisting of cationic and hydrophobic amino acids resulting in overall positive charge and amphipathic structure which facilitate its interaction with the negatively charged cell membrane [15]. Because of a net negative charge in cell membrane of cancer cells compared with normal cells, anti-cancer polypeptide is preferentially toxic towards cancer cells [14]. Mastoparan (MP) is a selective and potent anti-cancer polypeptide, isolated from wasp venom and involved in inflammation process, lysis of cell membrane, degranulation of mast cell, release of histamine and neutrophil [7, 8]. It can be classified into two groups according to their mode of action: (i) those acting through lysis of the cell by formation of pore in the cell membrane, (ii) those acting via interaction with G-protein-coupled receptors resulting in activation of degranulation mechanisms and leading to numerous types of secretions depending on the target cell type. MP induces mitochondrial-dependent apoptosis in cancer cells with less toxicity in comparison with normal cell.

Alendronate sodium (ALS) is a potent inhibitor of farnesyl pyrophosphate synthase. The ALS belongs to a class of medications called bisphosphonate drug and is used for the treatment of osteoporosis [16, 17]. Nevertheless, researchers have reported that ALS could be used as a cytotoxic agent by inhibition of tumor growth and migration with synergistic effects [18]. Previous data already confirms a low risk of both bone metastases and cancer recurrence in postmenopausal women with early stage breast cancer (EBC) [19, 20]. To date, the exact molecular mechanisms of the anti-tumor activity of ALS remains unknown [21, 22].

The advancement in nanotechnology allowed the delivery of chemotherapeutic agents to the desired site at relatively higher levels. In the current work, a nanoconjugate ALS-MP formula was firstly prepared and subsequently examined for its potential in suppressing lung cancer cells. Box-Behnken response surface design was applied. ALS-MP nanoconjugates’ particle size, encapsulation efficiency and the release profile were determined. The optimized ALS-MP formula was investigated for its potential contribution in cytotoxicity, cell cycle, caspase 3 analyses and annexin V staining on A549 cells.

## Materials and methods

The ALS was obtained as kind gift from EIPICO. Pharmaceuticals (10th of Ramadan city, Egypt). MP was from Sigma Aldrich, St. Louis, MI, USA.

### Experimental design for optimization of ALS-MP nanoconjugates

Box-Behnken response surface design was employed for formulating ALS-MP nanoconjugates using Design-Expert software (Version 12, Stat-Ease Inc., Minneapolis, MN, USA). The statistical effects of independent variables, namely, MP: ALS molar ratio (X_1_), incubation time (X_2,_ min), and sonication time (X_3_, min) on the observed response particle size (Y) were studied. The levels of the investigated factors are depicted in Table 1. According to the design, 15 experimental trials were generated by the software, including three center points.

**Table 1:** Independent variables’ levels and response constraint used in the Box-Behnken design for the optimization of ALS-MP nanoconjugates.

Independent variables	Levels		
	(-1)	(0)	(+1)
**X1: MP: ALS molar ratio**	1:1	1:5.5	1:10
**X2: Incubation time (min)**	10	35	60
**X3: Sonication time (min)**	3.0	6.5	10.0
**Responses**	Desirability constraint		
**Y1: Particle size (nm)**	Minimize		

**Abbreviations**: ALS, Alendronate sodium; MP, Mastoparan peptide.

The mean measured particle size for experimental runs as well as the levels of the variables used in the corresponding runs are displayed in Table 2. The best-fitting sequential model for the particle size data was selected based on the model fit statistical results. The model showing the greatest adjusted and predicted R^2^ and the least predicted residual sum of squares (PRESS) was used to represent the relation between the variables and the response. 2D-contour plots were generated by the software to display the influence of the studied factors and the interaction between them.

**Table 2:** Variables levels and observed response (particle size) for ALS-MP nanoconjugates experimental runs formulated according to Box-Behnken design generated.

Experimental run	Independent variables			Dependent variables
	MP: ALS molar ratio	Incubation time (min)	Sonication time (min)	Particle size (nm)
**F1**	**1:10**	10	6.5	291.6±2.3
**F2**	**1:5.5**	35	6.5	222.5± 3.5
**F3**	**1:10**	35	10.0	315.8±10.3
**F4**	**1:1**	60	6.5	181.9±12.3
**F5**	**1:1**	35	10.0	143.2±9.3
**F6**	**1:5.5**	10	3.0	218.5±10.3
**F7**	**1:1**	35	3.0	164.7±8.3
**F8**	**1:5.5**	60	10.0	241.8±10.3
**F9**	**1:10**	35	3.0	322.1±9.5
**F10**	**1:5.5**	35	6.5	221.3±.11.2
**F11**	**1:1**	10	6.5	133.9±10.3
**F12**	**1:5.5**	35	6.5	222.4±12.4
**F13**	**1:5.5**	60	3.0	268.6±9.4
**F14**	**1:5.5**	10	10.0	210.3±15.3
**F15**	**1:10**	60	6.5	343.4±18.3

### Preparation of ALS-MP nanoconjugates

ALS-MP nanoconjugates were prepared using the formulation parameters in the experimental runs shown in Table 2, generated based on the Box-Behnken experimental design. ALS and MP are dissolved, in various proportions according to the design, in 20 milliliters of deionized water. The prepared solutions were incubated and sonicated based on the specified times indicated in Table 2 according to the experimental design [23].

### Optimization of ALS-MP nanoconjugates

The examined independent variables were optimized by numerical method following the desirability function approach. The optimization aims to primarily minimize the size of the formulated ALS-MP nanoconjugates. Nonetheless, the predicted optimized formulation was prepared for further characterization.

### Particle size, zeta potential and thermodynamic stability determination

ALS-MP nanoconjugates’ particle size, polydispersity index and zeta potential were determined by appropriate dilution in double distilled water using a Zetasizer Nano ZSP particle size analyzer instrument (Malvern, UK).

The optimized ALS-MP was subjected to three freeze‒thaw cycles at −20 °C and +25 °C (12 h each). The optimized formula was then inspected for particle size determination using the same procedure described.

### *In vitro* release study

To determine the release profile of optimized ALS-MP nanoconjugates in comparison to ALS solution, 2 ml of prepared formulation and ALS solution were kept in the separate dialysis bag (molecular weight cut-off 12 kDa). Then tightly sealed dialysis bags were immersed in the 500 mL PBS (pH 7.4) at 37 °C with gentle agitation. At a fixed time interval, a 1 mL sample was then collected from the PBS medium, and the same amount of fresh PBS was added instantly. Thereafter collected samples were quantified spectrophotometrically at 287 nm and cumulative percentage drug released was obtained [24].

### Cytotoxicity of optimized ALS-MP nanoconjugates

The cytotoxicity efficacy of optimized ALS-MP nanoconjugates was performed on the A549 cell line using MTT assay. A549 cells were cultured in a Roswell Park Memorial Institute (RPMI) 1640 Medium supplemented with 10% fetal bovine serum (FBS), penicillin, and streptomycin. The cell line was grown at 37 °C under a humidified atmosphere with 5% CO2 to 80–90% confluence. The human tumor cell line A549 (adenocarcinomic human alveolar basal epithelial cells) used in this study was obtained from the VACSERA (Giza, Egypt) cell culture unit that was originally acquired from ATCC (Manassas, VA, USA).

For this experiment, A549 cells were grown in 96 well plates at the density of 5×10^3^ cells per well and incubated overnight. After stabilization, cells were treated with ALS-raw, MP-raw, and ALS-MP nanoconjugates and incubated for 24 h. Then previously treated cells were further treated with 5.0 mg/mL MTT solution (10 μL) then incubated for 4 h at 37 °C. Additionally, the collected supernatant was dispersed in 100 mL of DMSO to solubilize the formazan crystal. Samples were analyzed employing a microplate reader at 570 nm. Studies were carried out in triplicate [25].

### Cell cycle analysis

To analyze the effects of samples on the cell cycle, the flow cytometry method was utilized. The cells were treated with various sample formulations: ALS-raw, MP-raw, and ALS-MP nanoconjugates, and incubated for 24 h. After completion of incubation, cells were separated by centrifugation and fixed with 70% cold ethanol. Prior to washing of samples with PBS, samples were again separated by centrifugation. Separated cells were further stained with propidium iodide and RNAse before starting flow cytometry analysis [26, 27].

### Analysis of apoptosis by Annexin V staining

In order to analyze the comparative apoptotic activity of ALS-raw, MP-raw, and ALS-MP, the Annexin V method was implemented. For this purpose, A549 cells were grown in 6 well plates at the density of 1×10^5^ cells per well then incubated overnight with IC_50_ concentration of samples for 24 h at 37 °C. All samples were then centrifuged at 200×g for 5 min, and collected cells were resuspended in PBS at room temperature after dual washing. Further, 10 μL Annexin V and 5 μL propidium iodide solution supernatant were dispersed in the previously prepared samples and incubated at 25 °C for 5 min. Final samples were analyzed using a flow cytometer (FACS Calibur, BD Bioscience, CA, USA) in triplicate [28, 29].

### Analysis of Caspase 3

The Caspase 3 determination was carried out through the Caspase 3 Colorimetric Assay Kit (BioVision, Milpitas, CA, USA). In this case, A549 cells were grown in the density of 3×10^3^ cells per well and treated with control, ALS-raw, MP-raw, and ALS-MP nanoconjugates. Then samples were resuspended in ice-chilled lysate buffer and incubated in an ice medium for 10 min before centrifugation (10,000×g for 1 min). The analysis method for the Caspase 3 assay was carried according to the instructions of the manufacturer, and the developed color was determined by a microplate reader at 405 nm [27, 30].

### Statistical analysis

Data of the current study are expressed as the mean ± standard deviation (SD) following triplicate experimentation. The significance of the study was determined using Analysis of variance (ANOVA) followed by Tukey’s post hoc test. The p-value<0.05 represented the statistical significance of the data obtained. Statistical analysis was performed using GraphPad Prism8 (GraphPad Software Inc., San Diego, CA, US).

## Results

### Fit and diagnostic analysis

Amongst the explored sequential models, the best fitting model for the particle size of the developed ALS-MP nanoconjugates was found to be the quadratic model as indicated by its greatest correlation (R^2^) and least predicted residual sum of square (PRESS); results of the model fit analysis are displayed in Table 3.

**Table 3:** Model fit statistics for the particle size of ALS-MP nanoconjugates.

Source	SD	R^2^	Adjusted R^2^	Predicted R^2^	PRESS
Linear	7.97	0.9880	0.9847	0.9808	1118.31
2FI	8.34	0.9904	0.9833	0.9765	1366.96
Quadratic	3.59	0.9989	0.9969	0.9824	1021.50

Abbreviations: ALS, Alendronate sodium; MP, Mastoparan peptide; SD, standard deviation; PRESS, predicted residual error sum of squares; 2FI, two-factor interaction.

The adequate precision value was computed using the Deisgn Expert software to be 70.89. The adequate precision represents signal-to-noise ratio. It compares the range of the predicted values at the design points to the mean prediction error. A ratio exceeding 4 is desirable as it indicates appropriate model discrimination, i.e. the model has a strong enough signal to be used for optimization. Accordingly, the curernt adequate precision value ensures the suitability of the model to explore the experimental design space [31]. Diagnostic plots for particle size, developed for assessing the goodness of fit of the selected sequential model, are presented in Fig 1.

**Fig 1:** Diagnostic plots for particle size of ALS-MP nanoconjugates: (A) Box-Cox for power transforms, (B) externally studentized residuals vs. predicted particle size, (C) ex-ternally studentized residuals vs. run number, and (D) predicted vs. actual particle size. Abbreviations: ALS, Alendronate sodium; MP, Mastoparan peptide.

In Fig 1A that represents the Box-Cox plot for power transforms, the most appropriate lambda (λ) value of 1.05 (illustrated by the green line) lies within the 95% confidence interval for λ (-0.15 to 2.52, illustrated by red lines) indicating the absence of need for data transformation. The externally studentized residuals vs. predicted response and the residual vs. run plots presented in Fig 1B and 1C respectively, display randomly scattered points within the limits; this implies that there is neither constant error nor lurking variable that could interfere with the measured response [32]. Furthermore, the predicted vs. actual particle size plot (Fig 1D) shows good analogy between the predicted and measured particle size values, thus, assuring the model validity [27].

### Influence of variables on particle size (Y)

ALS-MP nanoconjugates exhibited nanosized formulations ranging from 143 to 343 nm as outlined in Table 2. As per the analysis of variance (ANOVA) results, the computed F-value of 500.55 (P < 0.0001) verified the validity of the nominated quadratic model with only a 0.01% probability that this value could be high owing to noise. The equation representing the quadratic model was given as follows in terms of coded factors:

$$\text{Y}=221.67+81.25{\;\text{X}}_{1}+22.63{\;\text{X}}_{2}–7.88{\;\text{X}}_{3}+1.00{\;\text{X}}_{1}{\text{X}}_{2}+3.50{\;\text{X}}_{1}{\text{X}}_{3}–4.75{\;\text{X}}_{2}{\text{X}}_{3}+8.45{\;\text{X}}_{1}^{2}+6.79{\;\text{X}}_{2}^{2}+5.79{\;\text{X}}_{3}^{2}$$

All linear (X_1_, X_2_, and X_3_) and quadratic (${\text{X}}_{1}^{2}$, ${\text{X}}_{2}^{2}$, and ${\text{X}}_{3}^{2}$) terms corresponding to the explored factors exhibited a significant impact on particle size (P < 0.0001 for the three linear terms, P = 0.0060, 0.0150, and 0.0268 for ${\text{X}}_{1}^{2}$, ${\text{X}}_{2}^{2}$, and ${\text{X}}_{3}^{2}$, respectively). In addition, the interaction term between the incubation and sonication times (X_2_X_3_) was also significant (P = 0.0456). Fig 2 demonstrates the three-dimensional (3D) surface plots and the two-dimensional (2D) contour plots for the effects of the investigated factors on the particle size and the interaction between them.

**Fig 2:** Response 3D-plots (A-C) and contour 2D-plots (D-F) for the influence of ALS:MP molar ratio (X1), incubation time (X2), and sonication (X3) on the particle size of ALS-MP nanoconjugates.

It was evident that both MP: ALS molar ratio and incubation time showed direct relationship with the particle size, while the sonication time showed inverse relationship. Accordingly, the particle size increases at higher MP level and incubation time, while at higher sonication times it decreases. This observation is confirmed by the positive sign of both X1 and X2 coefficients and the negative sign of X3. As per the value of the coefficients presented in the sequential model equation, the effect of variables can be ordered as follows: MP: ALS molar ratio > incubation time > sonication time. It is worthy to note that that the effect of the sonication time on size although being significant, yet it is the minimal amongst the investigated variables, so this effect may not be quite clear in Fig 2 as it represent the interaction between variables and not the individual effects. The figure showing the individual effect of variables is shown as (S1 Fig).

### Optimization

According to the previously set goal for producing nanoconjugates of minimized particle size, the optimized levels of the investigated factors were anticipated with an overall desirability of 0.991 in order to reach the desired formulation. The predicted levels for the optimized ALS-MP according to the design were 1:1 for MP: ALS molar ratio, 12.1 minutes for incubation time, and 9.1 minutes for sonication time. The formulation was prepared using the predicted optimized variables levels and further assessed for particle size and biological activity in cancer cells. The low percentage error of 1.55% between the predicted (132.85 nm) and observed particle size (134.91 ± 5.1 nm) indicates the validity of the optimization process.

The zeta potential value of the developed optimized ALS-MP was +18.87 ± 0.231 mV. The PDI of the optimized ALS-MP was 0.276 indicating a relatively homogeneous size. In addition, The optimized ALS-MP showed good thermodynamic stability with no significant variations in particle size after and before the three freeze‒thaw cycles.

### *In vitro* release study

The comparative *in vitro* release profile between ALS-MP nanoconjugates and ALS-raw was established. Outcomes of *in vitro* release study clearly revealed sustained release of ALS from the nanoconjugates. Contrastingly, in terms of percent cumulative release, a fast release of ALS was observed from conventional ALS suspension (Fig 3). Fig 3 demonstrated 41.2±8.6% cumulative release of ALS from conjugated formulation, and simultaneously 93±5.3% ALS was released from conventional suspension within 4 h. During study duration, conjugated formulation released almost all ALS load within 12h compared.

**Fig 3:** The in vitro release pattern of drug from optimized ALS-MP and ALS-raw.

### Cytotoxicity study

In order to obtain IC50 of different samples, a comparative cytotoxicity study was performed, and the result is depicted in Fig 4. The novel ALS-MP demonstrated the lowest IC50 (1.3 ± 0.34 μM) in comparison to ALS-Raw (37.6 ± 1.79 μM). Thus, the results indicated that when ALS was conjugated with MP, the IC50 of ALS was reduced significantly (p< 0.05).

**Fig 4:** Comparative cytotoxicity of various samples in terms of IC50. *Significantly different from Staurosporine p<0.05, #significantly different from MP p<0.05, $signifi-cantly different from ALS p<0.05.

### Cell cycle analysis

The effect of various formulations/samples such as control, MP, ALS-Raw, and ALS-MP on cell cycle was performed. Outcomes of the study clearly demonstrated a significantly higher percentage of cells in the G2-M phase after treatment with MP which found to be 25.48± 0.91% in comparing with 14.96 ±0.1 and 6.47±0.1 for ALS and ALS-MP, respectively (Fig 5). While increased cell population in pre G1 phase to be 28.47. ± 0.46%, while ALS was 12.61 ± 0.69. Relative to the control values, exposure of A549 cells to the ALS-MP resulted in significant cell death, as indicated by the 1305% increase in pre-G cell population.

**Fig 5:** Effect of various formulations on cell cycle. *Significantly different from control p<0.05, #significantly different from MP p<0.05, $significantly different from ALS-Raw p<0.05.

### Outcomes of Annexin V staining

The apoptotic study of various samples was carried out by flow cytometry after staining by Annexin V. Outcomes of apoptosis study demonstrated that formulation remarkably accelerated early, total, and in necrotic cell apoptosis compared to control, MP and ALS-Raw (Fig 6). Whereas maximum late apoptosis was exhibited by ALS-Raw formulation. It can be seen from Fig 6 that exposure of ALS-MP within the novel formulation significantly induced apoptosis (32.92± 0.96%), when compared to the untreated control (2.18%), ALS (12.61±0.82%), or MP (28.47±0.03%).

**Fig 6:** Determination of cellular mortality after Annexin V staining by flow cytometry. *Significantly different from control p<0.05, #significantly different from MP p<0.05, $sig-nificantly different from ALS-Raw p<0.05.

### Analysis of Caspase 3

The result of Caspase 3 analysis clearly exhibited ALS conjugated MP significantly increased the Caspase 3 quantity in treated cells as compared to ALS-Raw (Fig 7). Besides, MP also demonstrated an increment in the amount of Caspase 3 as compared to the control group. ALS-MP showed an increase of about 639%, compared to the increase of 209.1% and 209.2% induced by the MP and ALS, respectively.

**Fig 7:** Comparative effects of ALS-MP on Caspase 3. *Significantly different from control p<0.05, #significantly different from MP p<0.05.

## Discussion

Globally, among both men and women, lung cancer is by far the leading cause for cancer-related deaths [33]. According to previously reported database from world health organization (WHO), global estimates for the total mortality rate for lung cancer was (17%), followed by stomach cancer (12%), liver (9%), colon and rectum (9%), and breast cancer (7%) [34]. In the developed countries, lung cancer incidence and mortality rates are regarded the highest [35]. Interestingly, with the development of nanotechnology, nanocomplexes and nanocarriers has greatly aided the targeted delivery of high levels of chemotherapeutic agents to the desired site [36]. In this study, MP was used as carrier for ALS to improve cellular penetration ability of ALS and to improve its efficacy.

The experimental design results showed that both MP: ALS molar ratio and incubation time exhibited positive effect on the particle size, whereas the sonication time exhibited a negative effect. Increased particle size at higher drug levels in drug/polymer nanoconjugates has been previously reported [37, 38]. Increasing particle size along with increasing incubation time could possibly be attributed to increasing the liability of ALS conjugation with MP. Thus, as the incubation time increases, the number of drug molecules attaching to the peptide could probably increase leading to higher particle size of the formed nanoconjugates [39]. Moreover, previously published studies have indicated the negative effect for the sonication time on the particle size for various nanoparticulate systems [40, 41]. This could be owing to the cavitation forces developed by the ultrasonic waves of the sonicator. These forces might cause particle size reduction by virtue of possible fractionation of the agglomerated nanoconjugate clusters [42, 43]. A minimized particle size of the prepared ALS-MP formula was achieved as a result of the application of experimental design in drug formulation. Box-Behnken design utilized the data from the experimental runs (with the variable factor levels) in order to achieve the optimized formula with minimum particle size of 134.91± 5.1 nm. According to recent studies carried out on anti-cancer therapeutics, nanotechnology-based pulmonary drug delivery systems holds a great potential in improving retention of anti-cancer drugs in the lung in addition to the demonstrated limiting of its penetration into the blood stream, thus minimizing chemotherapy-related unwanted adverse effect [6, 44, 45]. Of note, the size of particulate delivery systems is proved to be an influential parameter that could greatly affect the penetration of active ingredients across the biological membranes [45].

ALS exerts its antiproliferative effects via induction of apoptosis and cell cycle arrest. Similar cytotoxic effects were also observed with MP; therefore, it would be a good candidate to improve the activity of ALS against lung cancer [46, 47] novel ALS-MP formula developed in this study showed significant cytotoxicity against the A549 lung cancer cells. This novel formula significantly decreased the IC50 of ALS by more than 90%, indicating that the ALS-MP nanocomplexes act as an effective delivery system for ALS.

These results are consistent with the cytotoxic activity of ALS in human lung cancer cell lines [14]. The improved cytostatic activity of ALS formula could be attributed to the enhanced permeability of the novel formulation. Free ALS is passively transported across the cell membrane, whereas, while ALS incorporated into the MP appears to be internalized via endocytosis. Furthermore, MP are known to facilitate the delivery of amphiphilic agents across the lipid rich bio-membrane of cells, hence increasing their intracellular concentrations [48, 49].

The apoptotic activity of ALS when incorporated ALS-MP was found to be significantly enhanced relative to the plain formula and free ALS. It appears that ALS -MP affected cell population in the different phases of cell cycle. This novel nanocarrier platform loaded with ALS increased the percentage of cells in the S and pre-G1 phases while decreasing the population of cells in the G2-M phase. G1-phase arrest of cell cycle progression highlights the apoptotic potential of the novel ALS formulation developed in this study. In accordance with these findings, it has been previously shown that ALS treatment induces apoptosis in human lung adenocarcinoma cells [32, 50]. Yet, the ALS-MP has improved the apoptotic activity of ALS significantly higher than the levels associated with the free drug. The increased apoptotic activity of the ALS formula might be due to enhanced membrane penetration capacity of ALS. This is in agreement with reports in the literature showing that structural modifications of ALS to enhance its cellular internalization resulted in apoptosis and cell cycle arrest in the S phase colorectal cancer cells [51, 52]. In addition, we found that ALS significantly increased the population of cells in the pre-G phase which is consistent with other reports in the literature [53]. These findings were confirmed by apoptosis analysis using annexin V, where the novel ALS formula was found to significantly increase early, late, and total cell death. This is in agreement with previous findings in the literature highlighting the importance of apoptosis in the anti-proliferative properties of ALS [54]. This increase in apoptosis associated with the ALS formula could be due to the penetration nature of the MP which can confer improved delivery of ALS to its site of action [55].

ALS-MP also significantly increased the mRNA expression of caspase 3, which is consistent with reports in the literature highlighting the potential of ALS to upregulate cellular caspase 3 activity [56]. It is also known that ALS-MP the targeting and proapoptotic activity of active drugs including their effects on cleaved caspase-3 content in A543 cells. changes in the expression of p53 and the Bcl2 family of proteins are known to induce apoptosis and cell cycle arrest in stressed cells [57–59].

## Conclusions

In the present study, the Box-Behnken design was utilized to optimize ALS-MP formula. The optimized ALS-MP exhibiting a minimal particle size, further showed a gradual and complete *in vitro* release when compared with raw ALS. Nonetheless, the *in vitro* experiments carried out on A549 cells clearly demonstrated that the optimized formula ALS-MP had significantly improved the parameters related to the cytotoxic activity towards cancerous cells, amongst which a lower IC50, the obvious enhancement of anti-proliferative activity, the increase of apoptosis and necrosis cell populations. Thus, it can be concluded that the remarkable favorable results for ALS-MP nanoconjugate, making it a novel treatment approach against lung cancer.

## Supporting information

S1 Fig The figure showing the individual effect of variables. (PNG)
